The article "Prosthetic shape, but not stiffness or height, affects the maximum speed of sprinters with bilateral transtibial amputations" was retracted in 2022. Reasons: errors in the analysis; unreliable results or conclusions; concerns about the data; concerns about the results or conclusions.

# Prosthetic shape, but not stiffness or height, affects the maximum speed of sprinters with bilateral transtibial amputations

**DOI:** 10.1371/journal.pone.0229035

**Published:** 2020-02-20

**Authors:** Paolo Taboga, Owen N. Beck, Alena M. Grabowski

**Affiliations:** 1 Department of Kinesiology, California State University, Sacramento, California, United States of America; 2 The George W. Woodruff School of Mechanical Engineering, Georgia Institute of Technology, Atlanta, Georgia, United States of America; 3 School of Biological Sciences, Georgia Institute of Technology, Atlanta, Georgia, United States of America; 4 Department of Integrative Physiology, University of Colorado, Boulder, Colorado, United States of America; 5 Department of Veterans Affairs, Eastern Colorado Healthcare System, Aurora, Colorado, United States of America; Holland Bloorview Kids Rehabilitation Hospital, CANADA

## Abstract

Running-specific prostheses (RSPs) have facilitated an athlete with bilateral transtibial amputations to compete in the Olympic Games. However, the performance effects of using RSPs compared to biological legs remains controversial. Further, the use of different prosthetic configurations such as shape, stiffness, and height likely influence performance. We determined the effects of using 15 different RSP configurations on the maximum speed of five male athletes with bilateral transtibial amputations. These athletes performed sets of running trials up to maximum speed using three different RSP models (Freedom Innovations Catapult FX6, Össur Flex-Foot Cheetah Xtend and Ottobock 1E90 Sprinter) each with five combinations of stiffness category and height. We measured ground reaction forces during each maximum speed trial to determine the biomechanical parameters associated with different RSP configurations and maximum sprinting speeds. Use of the J-shaped Cheetah Xtend and 1E90 Sprinter RSPs resulted in 8.3% and 8.0% (p<0.001) faster maximum speeds compared to the use of the C-shaped Catapult FX6 RSPs, respectively. Neither RSP stiffness expressed as a category (p = 0.836) nor as kN·m^-1^ (p = 0.916) affected maximum speed. Further, prosthetic height had no effect on maximum speed (p = 0.762). Faster maximum speeds were associated with reduced ground contact time, aerial time, and overall leg stiffness, as well as with greater stance-average vertical ground reaction force, contact length, and vertical stiffness (p = 0.015 for aerial time, p<0.001 for all other variables). RSP shape, but not stiffness or height, influences the maximum speed of athletes with bilateral transtibial amputations.

## Introduction

Athletes with bilateral transtibial amputations (TTAs) who use running-specific prostheses (RSPs) have achieved Olympic-qualifying 400 m performances [1] and have won professional races competing against non-amputee elite athletes [2]. RSPs are comprised of carbon fiber and can store and return elastic energy, but do not fully function like biological legs [3–5]. Due in part to the different biomechanics elicited by athletes with TTAs using RSPs compared to non-amputees [6], (e.g. lower stance average vertical ground reaction force (GRF) and longer ground contact time), the governing body of track and field, the International Association of Athletics Federations (IAAF), mandates that athletes with TTAs must prove that their use of RSPs does not provide a performance advantage compared to non-amputees (IAAF Rule 144.3, [7]). The configuration of an RSP (shape, stiffness and height) likely affects the performance of athletes with TTAs [5, 8] and must comply with International Paralympic Committee (IPC) regulations [9] for athletes to participate in official races. It is therefore of paramount importance for fair competition that the rules and regulations governing athletics are based on empirical scientific evidence.

There are many biomechanical variables that influence maximum speed and running performance [10]. Running speed equals the product of step frequency and step length, where a step consists of ground contact and the subsequent aerial time. To achieve faster speeds, sprinters typically increase both step frequency and step length [11, 12]. Step length can be calculated as the product of contact length (L_c_) (the distance travelled by the center of mass during ground contact) and stance average vertical GRF relative to body weight. Thus, running speed also equals the product of L_c_, stance average vertical GRF, and step frequency [12]. Among these factors, sprinters achieve faster speeds by increasing stance average vertical GRF [12] and step frequency, and reducing ground contact time (t_c_) [12, 13]. Elite non-amputee sprinters have reached maximum speeds of up to 10.2 m·s^-1^ during 40 m sprint trials over ground [11], and up to 11.7 m·s^-1^ during brief treadmill sprints (20 steps) [12].

Use of RSPs has enabled athletes with TTAs to achieve remarkable sprinting speeds [1, 14, 15]. In particular, previous studies have reported a maximum speed of 10.8 m·s^-1^ for a sprinter with bilateral TTAs [1] and 11.55 m·s^-1^ for a sprinter with a unilateral TTA during brief treadmill sprints [16]. Similar to non-amputees, athletes with unilateral and bilateral TTAs who use RSPs achieve faster running speeds by increasing step length, step frequency, stance average vertical GRF relative to body weight and contact length [3–5]. Increased step frequency occurs from decreasing both contact time [3–5] and aerial time [1]. However, when running at maximal or near-maximal speeds, athletes with unilateral and bilateral TTAs who use RSPs generate lower stance average vertical GRFs [1, 3, 5] and have longer [17] or similar [5] contact times in their affected legs compared to non-amputees, which likely limits their maximum sprinting speed [1, 3]. It is not clear how aerial time affects maximum speed: previous studies have reported aerial times that are either shorter [1] or longer [3, 4] in the affected legs of athletes with TTAs using RSPs compared to the biological legs of non-amputees.

The sprinting ability of athletes with TTAs may be limited by the stiffness of their RSPs. Unlike biological legs, the mechanical characteristics of RSPs, such as stiffness, cannot be actively modulated during running. Previous studies have found that to achieve faster running speeds, non-amputees increase vertical stiffness (k_vert_) [18], while either keeping leg stiffness (k_leg_) constant [19] or increasing it [4]. RSPs are passive-elastic springs that have curvilinear (quadratic) force-displacement profiles, where the greater the magnitude of compression, the greater the stiffness of the RSP [20]. Manufacturers of RSPs assign a stiffness category to each prosthetic model, from 1 (less stiff) up to ~9 (more stiff) depending on the model [21–23]. An athlete with a TTA is prescribed a prosthetic stiffness category based on his/her body mass and, for some manufacturers, activity type (short- vs. long- distance running). Larger/heavier athletes are prescribed greater stiffness categories compared to smaller/lighter athletes [21–23]. However, across manufacturers the recommended stiffness categories do not necessarily elicit the same stiffness values for a given athlete’s body mass [20].

McGowan et al. [4] found that sprinters with unilateral and bilateral TTAs increased dimensionless vertical stiffness (K_vert_), but decreased dimensionless leg stiffness (K_leg_) in their affected legs at faster speeds. However, non-amputees increased K_vert_ and K_leg_ at faster running speeds. Across speeds ranging from 3 to 9 m·s^-1^, RSP stiffness affects the biomechanics of sprinters with bilateral TTAs [5]. Use of stiffer RSP categories elicits greater peak and stance average vertical GRFs, increases k_leg_ and decreases t_c_ compared to use of less stiff RSPs, suggesting that more stiff RSP categories may permit increased K_vert_ and K_leg_ and thus elicit faster maximum sprinting speeds in athletes with bilateral TTAs. However, the effects of prosthetic stiffness on the biomechanical variables that determine running speed are mitigated at progressively faster speeds [5]. Particularly at faster speeds (>7 m·s^-1^), the differences in stance average vertical GRFs and t_c_ between more stiff and less stiff RSPs are modest. Thus, it is unclear if prosthetic stiffness affects the maximum speeds of athletes with bilateral TTAs.

RSPs mimic the spring-like behavior of tendons and ligaments during running by storing elastic energy during the first half of the contact phase and returning most of this energy during the second half of the contact phase [6, 20, 24]. In non-amputees, the storage and release of elastic energy in the Achilles tendon is described by Mero et al. [10] as a “force performance potentiation” that allows non-amputee sprinters to apply greater forces on the ground at progressively faster speeds. Kubo et al. [25] calculated that the elastic energy returned by tendons contributes up to 42% of the total mechanical work performed during fast dorsi/plantarflexion cycles (average joint rotation speed: 60 deg·s^-1^). Others [26] claim that the dynamics of force development by the muscles determine the amount of mechanical work performed, not the amount of stored elastic energy during stretch-shortening cycles. Thus, it is not clear how use of RSPs with different stiffnesses affects force production and elastic energy storage and return in athletes with TTAs.

Tendon and RSP hysteresis, defined as the percentage of elastic energy lost during recoil relative to the energy stored during loading [20], affects the magnitude of elastic energy return during running and sprinting. Previous studies that have measured *in-vivo* Achilles tendon hysteresis in non-amputees report values between 6.8% [27] and 30% [28], while *in-vitro* measurements of mammalian tendons report hysteresis between 7% [29] and 10% [30]. The hysteresis of an RSP, fitted with a rubber sole provided by each manufacturer and measured using a materials testing machine, ranges from 4.3% (J-shaped RSPs, Fig 1B and 1C) to 5.1% (C-shaped RSPs, Fig 1A) [20]. All of these hysteresis values suggest that a non-trivial portion of energy is lost in each step during running in tendons and in the RSPs used by athletes with TTAs. Different hysteresis values among RSP models [20] affect the relative amount of energy returned in each step [24] and may therefore influence sprinting performance in athletes with TTAs.

**Fig 1:** Three RSP models used in the study. **a)** Freedom Innovations Catapult FX6 (C-shaped) configured 2 cm taller than the International Paralympic Committee maximum allowable height (IPC max), **b)** Össur Flex-Foot Cheetah Xtend (J-shaped) configured at the IPC max and **c)** Ottobock 1E90 Sprinter (J-shaped) configured 2 cm shorter than the IPC max.

Running performance may also be influenced by leg length. Hypothetically, longer legs could allow athletes to achieve longer steps and, for a given step frequency, faster speeds. Athletes with bilateral TTAs can alter their leg lengths by changing the height of their RSPs. However, these athletes must adhere to the International Paralympic Committee (IPC) guidelines [9, 31] to compete in sanctioned track and field events. These guidelines set a maximum standing body height (MASH) for each athlete based on their intact limb dimensions, thereby limiting the maximum height of their RSPs. Previously, we [5] found that increasing prosthetic height by 2 cm increased contact length by 2.3 cm, but decreased step frequency by 0.021 Hz compared to the IPC maximum height across speeds of 3 to 9 m·s^-1^. Slower step frequencies may be due to the greater rotational moment of inertia of the whole leg and possibly negate any effect of prosthetic height on maximum running speed. Yet, though we previously reported step frequency and step length for speeds of 3 to 9 m·s^-1^, it is not clear if this negative correlation between step length and step frequency due to height is retained at maximum sprinting speeds.

We determined the maximum speeds elicited by athletes with bilateral TTAs using 15 different RSP configurations (models, stiffness, and heights). First, we hypothesized that use of stiffer RSPs (greater category and kN·m^-1^) would allow faster maximum sprinting speeds in athletes with bilateral TTAs compared to use of more compliant RSPs (lower category and kN·m^-1^). Second, we hypothesized that use of taller RSPs would allow athletes to achieve faster maximum sprinting speeds compared to use of shorter RSPs. Third, we hypothesized that the RSP configuration that allows athletes to achieve faster maximum sprinting speeds would be associated with greater stance-average vertical GRF, longer contact length, and shorter ground contact time. Lastly, we hypothesized that the RSP configuration that allows the fastest maximum speed would be associated with the greatest mechanical energy return per step.

## Materials and methods

### Subjects

Five male athletes with bilateral transtibial amputations (age: 24.8 ± 4.8 years) participated and were the same subjects as in Beck et al. [5, 24]. All participants had at least one year of experience running using their own RSPs and competed in sanctioned track and field races (Table 1). The experimental protocol was approved by the Colorado Multiple Institutional Review Board (COMIRB #13–2315) and the USAMRMC Office of Research Protection, Human Research Protection Office. All subjects gave informed written consent according to the COMIRB and USAMRMC.

**Table 1:** Demographic and anthropometric data of subjects with bilateral transtibial amputations.

Subject	Age (yrs)	Mass (kg)	Cause of Amputation	Primary event(s)	Usual RSP model	IPC Max height (m)	IPC Max L_0_ (m)	1E90 Sprinter L_0_ (m)	Cheetah Xtend L_0_ (m)	Catapult FX6 L_0_ (m)
**1**	25	69.3	Congenital	100 m / 200 m	Cheetah Xtend	1.80	0.97	0.97	0.97	1.07
**2**	23	76.3	Congenital	long jump	1E90 Sprinter	1.88	1.07	1.04	1.07	1.07
**3**	18	75.0	Congenital	100 m / 200 m	Cheetah Xtend	1.87	1.05	1.05	1.05	1.05
**4**	31	70.4	Trauma	400 m	Cheetah Xtend	1.90	1.10	1.10	1.10	1.10
**5**	27	70.5	Infection	5000 m	Flex-Run	1.87	1.06	1.06	1.06	1.06
**Average**	24.8	72.3				1.86	1.05	1.04	1.05	1.07
**S.D.**	4.8	3.1				0.04	0.05	0.05	0.05	0.02

Mass includes the athlete and their RSPs. Usual RSP model is the model used in competitions. Maximum International Paralympic Committee body height (IPC Max height) is the maximum allowable overall body height of each subject according to the IPC guidelines [31], L_0_ is leg length, measured from the greater trochanters to the most distal locations of the unloaded RSPs. The resulting Ottobock 1E90 Sprinter, Össur Flex-Foot Cheetah Xtend and Freedom Innovations Catapult FX6 prosthetic leg lengths represent the closest attainable maximum IPC-regulated leg lengths for each participant and prosthetic model combination. There were no statistically significant differences in L_0_ between RSP models or compared to the IPC Max L_0_.

### Experimental design

We used a repeated-measures experimental design. On the first day, each participant completed an alignment and accommodation session. During this session, a certified prosthetist aligned participants to three different RSP models (C-shaped Freedom Innovations Catapult FX6, Irvine, CA, USA; J-shaped Össur Flex-Foot Cheetah Xtend, Reykjavik, Iceland; J-shaped Ottobock 1E90 Sprinter, Duderstadt, Germany, Fig 1) at the manufacturer recommended stiffness category and maximum prosthetic height allowed by the IPC guidelines [31]. Each subject used two different sets of sockets: one set when running with J-shaped RSPs, and one set when running with C-shaped RSPs. The two sets of sockets were identical in terms of materials and overall shape/dimension, the only difference between sockets was the location and design of the RSP attachment (see Fig 1). Prosthetic height was adjusted by using different pylon lengths for the C-shaped Catapult FX6 model (Fig 1A) and by using a custom-made height-adjustment bracket for the J-shaped Cheetah Xtend and 1E90 Sprinter models (Fig 1B and 1C). A rubber sole was attached beneath the distal end of each RSP [20]. If the RSP model geometry and residual limb anatomy did not allow a participant to match the maximum IPC height at the time of testing [31], we selected the configuration that was as close as feasible to the maximum IPC competition height. For example, the height of an athlete with long residual limbs using C-shaped RSPs was greater than the IPC competition height and the height of an athlete with short residual limbs using J-shaped RSPs was shorter than the maximum IPC competition height. For each RSP model, each athlete initially ran on a treadmill at self-selected speeds, and provided feedback to the prosthetist who aligned and adjusted each RSP. Then subjects practiced progressively faster sprints on a 27 m runway covered with a rubber surface and on a treadmill until both the prosthetist and subject were satisfied with the alignment of the RSPs. The alignment and accommodation session lasted approximately 6–7 hours per participant.

On subsequent days, we asked participants to run over a range of speeds up to their maximum speed using three different RSP stiffness categories per model: manufacturer-recommended, and one category more stiff and one category less stiff than recommended. We randomized the trial order (three RSP models x three stiffness categories, nine trials). The stiffness category that elicited the fastest maximum speed for each RSP model was subsequently used with prosthetic heights that were increased or decreased by 0.02 m with respect to the maximum IPC height to determine the effects of prosthetic height on maximum speed. If the closest achievable height, based on an athlete’s residual limb lengths and the build height of the RSPs, was taller than the maximum IPC competition height, we increased prosthetic height by 0.02 m and 0.04 m. If the closest achievable height was shorter than the maximum IPC competition height, we decreased prosthetic height by 0.02 m and 0.04 m. In order to mitigate potential learning effects, we randomly inserted these trials into the trial order (three RSP models x two RSP heights = six trials). To minimize the potential for fatigue, we limited the maximum number of series of trials (from 3 m·s^-1^ to maximum speed) to three per day and, based on subject’s feedback, scheduled additional rest days between testing sessions. The duration of the testing protocol (fitting session, test sessions and rest days) was typically 10–11 days.

### Maximum speed determination

For each combination of RSP model, stiffness, and height, subjects performed a series of trials over a range of speeds. The initial speed was set at 3 m·s^-1^, and was incremented by 1 m·s^-1^ for each subsequent trial until subjects approached their maximum speed. Subsequently, smaller speed increments were employed until subjects reached their maximum speed [3]. We considered a trial to be successful if the subject could achieve at least 10 strides at the selected speed without moving backward on the treadmill. After a successful trial, subjects were allowed to rest for as much time as they needed before running at a faster speed. If the subject could not finish the trial, they were allowed to repeat that speed or select a slower speed (i.e. select a smaller increment from the last successful trial). The fastest trial was identified as the maximum speed for a given RSP configuration. We monitored the forward/backward movement of subjects on the treadmill with two reflective markers placed on each subject’s posterior superior iliac spines collected at 200 Hz by a 3D motion capture system (Vicon Nexus, Oxford, UK). The treadmill speed was monitored by tracking two reflective markers placed on the distal end of each RSP during the contact phase of the trials.

### Measurements and calculations

We collected GRFs at 1000 Hz on a 3D force measuring treadmill (Treadmetrix, Park City, USA). For each maximum speed trial, we used a custom MATLAB script (Mathworks Inc., Natick, MA, USA) to filter the GRFs using a fourth order Butterworth filter with a 30 Hz cutoff. We measured ground contact time (t_c_) and aerial time (t_a_), then calculated step frequency (f_Step_) and step length (l_step_). We measured peak and stance average vertical GRFs, and peak positive and negative horizontal GRFs and we calculated dimensionless stiffness, K_vert_ and K_leg_ [4]. We also calculated and mechanical power (P_RSP_, in W·kg^-1^) and energy return (E_RSP_, J·kg^-1^·m^-1^) during the second half of ground contact (see Appendix for detailed description of all measurements and calculations).

### Statistical analyses

We used a linear mixed model to determine the effects of RSP model, stiffness category, and height on maximum speed. We then used a second linear mixed model to determine the effects of RSP model, actual stiffness (in kN·m^-1^), and height on maximum speed. We used a third linear mixed model to determine the effects of contact and aerial times, peak and stance average vertical GRFs, peak positive and negative horizontal GRFs, and vertical and leg dimensionless stiffness on maximum speed. Step frequency and step length were excluded from this model given their intrinsic interaction with maximum speed (Eqs 1 and 2). For each of the three analyses, we obtained the final linear mixed model by iteratively removing all non-significant effects and interactions on maximum speed [32]. Then, we used five separate random effects linear models to evaluate the independent influence of step frequency, step length, hysteresis, prosthetic mechanical power, and prosthetic energy return on maximum speed. Lastly, interactions between RSP models and all parameters correlated with maximum speed were evaluated with post-hoc analyses using random effects linear models. We selected linear mixed models and random effects linear models, as opposed to simple linear regression analyses, in order to control for subject variability: each subject was classified as a random effect, while the independent variables were classified as fixed-effect variables. Linear mixed models and random effects linear models are particularly useful in repeated-measures designs [32], taking into account the lack of independence between observations within the same subject (e.g. the same subject using different RSP configurations) and also allowing for subjects missing some outcomes to be included in the analysis (e.g. if a subject cannot run on a specific RSP configuration due to the anatomy of his residual limbs). We carried out our statistical analyses using R-studio (Boston, MA) software. We also calculated the R^2^ value from the linear mixed models and random effects linear models according to Nakagawa and Schielzeth [33]. Significance was set at p<0.05. When applicable, we implemented Bonferroni corrections to account for multiple comparisons.

## Results

### Maximum speed and RSP configuration

We found a significant effect of RSP model on maximum speed. Subjects reached maximum speeds of 9.42 ± 0.90 m·s^-1^ (average ± SD) using the Össur Flex-Foot Cheetah Xtend RSPs, 9.31 ± 0.80 m·s^-1^ using the Ottobock 1E90 Sprinter RSPs and 8.68 ± 0.95 m·s^-1^ using the Freedom Innovations Catapult FX6 RSPs. While controlling for covariates, the use of the J-shaped Cheetah Xtend and 1E90 Sprinter RSPs facilitated 8.3% (p<0.001) and 8.0% (p<0.001) faster maximum speeds compared to use of the C-shaped Catapult FX6 RSPs, respectively. We found no significant differences in maximum speeds between the Cheetah Xtend and 1E90 Sprinter RSPs (p = 0.842). We found no effect of prosthetic stiffness when expressed as a category (p = 0.836, Fig 2A, Appendix Table 1), or when expressed in kN·m^-1^ (p = 0.916) on maximum speed. In addition, prosthetic height had no effect on maximum speed (p = 0.762, Fig 2B, Appendix Table 2).

**Fig 2:** **Average maximum speed as a function of: a) stiffness category (Rec is the recommended category) and b) change in prosthetic height (Δh) compared the International Paralympic Committee maximum allowable height (IPC max).** Error bars represent standard deviations. We found no effect of RSP stiffness category (p = 0.836) or height (p = 0.762) on maximum speed. Use of the J-shaped Cheetah Xtend and 1E90 Sprinter RSPs resulted in 8.3% and 8.0% faster maximum speeds, respectively, compared to the C-shaped Catapult FX6 RSPs (p<0.001).

### Biomechanical variables associated with maximum speed

We found that among all investigated biomechanical variables, contact time (t_c_), aerial time (t_a_), stance average vertical ground reaction force (GRF_avg,z_, in units of body weight, BW), and contact length (L_c_) together with leg and vertical dimensionless stiffness (K_leg_ and K_vert_) were associated with maximum speed:

$$\mathrm{Maximum}\;\mathrm{speed}\;\left(m\cdot s^{-1}\right)=‐68.11t_{c}‐5.77t_{a}+0.92{\mathrm{GRF}}_{\mathrm{avg},z}+7.83L_{c}‐0.02K_{\mathrm{leg}}+0.003K_{\mathrm{vert}}+7.67;\;(R^{2}=0.995)$$ (Eq 1)

For example, while controlling for covariates, a 0.01 second decrease in t_c_ was associated with a 0.68 m·s^-1^ faster maximum speed (p<0.001, Fig 3A), a 0.01 second decrease in t_a_ was associated with a 0.06 m·s^-1^ faster maximum speed (p = 0.015, Fig 3B), a 0.1 BW increase in GRF_avg,z_ was associated with a 0.09 m·s^-1^ faster maximum speed (p<0.001, Fig 3C), a 0.01 m increase in L_c_ was associated with a 0.08 m·s^-1^ faster maximum speed (p<0.001, Fig 3D), a one unit decrease in K_leg_ was associated with a 0.02 m·s^-1^ faster maximum speed (p<0.001, Fig 3E), and a one unit increase in K_vert_ was associated with a 0.003 m·s^-1^ faster maximum speed (p<0.001, Fig 3F). And, while controlling for covariates, a 1 m·s^-1^ faster maximum speed was associated with a 0.015 s decrease in t_c_ (12% shorter t_c_ compared to the average, p<0.001), a 0.173 s decrease in t_a_ (153% shorter, p = 0.015), a 1.09 BW increase in GRF_avg,z_ (57% greater, p<0.001), a 0.13 m increase in L_c_ (12% longer, p<0.001), a 50 unit decrease in K_leg_ (242% lower, p<0.001), and a 333 unit increase in K_vert_ (237% greater, p<0.001).

**Fig 3:** **Maximum speed as a function of: a) contact time (t**_**c**_**), b) aerial time (t**_**a**_**), c) stance average vertical ground reaction force (GRF**_**avg,z**_**), d) contact length (L**_**c**_**), e) dimensionless leg stiffness (K**_**leg**_**), and f) dimensionless vertical stiffness (K**_**vert**_**).** Each data point represents a single subject and RSP model. The dashed lines are regression lines obtained from Eq 1 (R^2^ = 0.995, see text) isolating each independent variable respectively: a) Maximum speed (m⋅s^−1^) = −68.11t_c_+17.08 (p<0.001), b) Maximum speed (m⋅s^−1^) = −5.77t_a_+9.80 (p = 0.015), c) Maximum speed (m⋅s^−1^) = 0.92GRF_avg,z_+7.41 (p<0.001), d) Maximum speed (m⋅s^−1^) = 7.83L_c_+0.89 (p<0.001), e) Maximum speed (m⋅s^−1^) = −0.02×K_leg_+9.53 (p<0.001), and f) Maximum speed (m⋅s^−1^) = 0.003×K_vert_+7.28 (p<0.001).

Using a post-hoc analysis, we found that at their respective maximum speeds, use of the Cheetah Xtend RSPs resulted in 5.0% and 5.1% shorter t_c_ compared to use of the 1E90 Sprinter and Catapult FX6 RSPs, respectively (p<0.001 for both comparisons). Use of the Catapult FX6 RSPs resulted in 6.9% shorter t_a_ compared to use of the Cheetah Xtend RSPs (p = 0.002), while there were no differences in t_a_ when using the Cheetah Xtend versus 1E90 Sprinter RSPs (p = 0.100) and the Catapult FX6 versus 1E90 Sprinter RSPs (p = 0.146). Use of the Cheetah Xtend RSPs resulted in 4.3% and 5.4% greater GRF_avg,z_ compared to use of the 1E90 Sprinter (p = 0.026) and Catapult FX6 (p = 0.027) RSPs, respectively. Use of the 1E90 Sprinter RSPs resulted in 4.0% longer L_c_ compared to use of the Cheetah Xtend RSPs (p<0.001), which in turn resulted in 3.1% longer L_c_ compared to use of the Catapult FX6 RSPs (p<0.001). Use of the 1E90 Sprinter RSPs resulted in 9.4% lower K_leg_ compared to use of the Cheetah Xtend RSPs (p = 0.02), which in turn resulted in 17.2% lower K_leg_ compared to use of the Catapult FX6 RSPs (p<0.001). Use of the 1E90 Sprinter RSPs resulted in 12% lower K_vert_ compared to use of the Catapult FX6 RSPs (p = 0.001), but K_vert_ was not different compared to use of the Cheetah Xtend RSPs (p = 0.118).

### The association of step length and step frequency on maximum speed

We found that across all RSP configurations, both step length (l_step_, Fig 4A) and step frequency (f_step_, Fig 4B) were correlated with maximum speed:

$$\mathrm{Maximum}\;\mathrm{speed}\;\left(m\cdot s^{-1}\right)=3.80\times l_{\mathrm{step}}+1.24;\;\left(R^{2}=0.843,\;p<0.001\right),$$ (Eq 2)

$$\mathrm{Maximum}\;\mathrm{speed}\;\left(m\cdot s^{-1}\right)=1.27\times f_{\mathrm{step}}+3.59;\;\left(R^{2}=0.463,\;p=0.002\right),$$ (Eq 3)

We found that use of the Cheetah Xtend and 1E90 Sprinter RSPs resulted in 9.0% longer l_step_ compared to use of the Catapult FX6 RSPs (p<0.001 for both comparisons). We found no differences in f_step_ between RSP models (p>0.599 for all comparisons).

**Fig 4:** **Maximum speed as a function of: a) step length (l**_**step**_**) and b) step frequency (f**_**step**_**).** Each data point represents a single subject and RSP model. The dashed line is the regression line obtained from Eq 2: Maximum speed (m⋅s^−1^) = 3.80×l_step_+1.24 (R^2^ = 0.843, p<0.001) and Eq 3: Maximum speed (m⋅s^−1^) = 1.27×f_step_+3.59 (R^2^ = 0.463, p = 0.002).

### The association of elastic energy return on maximum speed

We found that maximum speed was positively correlated with both prosthetic mechanical power return (P_RSP_, Fig 5A) and elastic energy return (E_RSP_, Fig 5B) across all RSP configurations:

$${\mathrm{Maximum}\;\mathrm{speed}\;(m\cdot s}^{‐1})=0.59\times P_{\mathrm{RSP}}+5.66;\;\left(R^{2}=0.597,\;p<0.001\right),$$ (Eq 4)

$${\mathrm{Maximum}\;\mathrm{speed}\;(m\cdot s}^{‐1})=0.51{\times E}_{\mathrm{RSP}}+7.71;\;\left(R^{2}=0.397,p=0.046\right),$$ (Eq 5)

**Fig 5:** **Maximum speed as a function of: a) RSP mechanical power return (P**_**RSP**_**), b) RSP mechanical energy return (E**_**RSP**_**), and c) hysteresis (H).** The dashed lines are the regression lines from Eq 4: Maximum speed (m⋅s^−1^) = 0.59×P_RSP_+5.66 (R^2^ = 0.597, p<0.001), Eq 5: Maximum speed (m⋅s^−1^) = 0.51×E_RSP_+7.71 (R^2^ = 0.397, p = 0.046) and Eq 6: Maximum speed (m⋅s^−1^) = −0.52×H+11.55 (R^2^ = 0.572, p<0.001).

Among all maximum speed trials, P_RSP_ ranged from 3.92 W·kg^-1^ (corresponding to an 8 m·s^-1^ maximum speed) to 8.22 W·kg^-1^ (corresponding to a 9.5 m·s^-1^ maximum speed), while E_RSP_ ranged from 2.11 J·kg^-1^·m^-1^ (corresponding to an 8 m·s^-1^ maximum speed) to 4.05 J·kg^-1^·m^-1^ (corresponding to a 9.5 m·s^-1^ maximum speed). Use of the 1E90 Sprinter RSPs resulted in 15.9% and 20.3% greater mechanical power return compared to use of the Catapult FX6 and Cheetah Xtend RSPs, respectively (p = 0.001 for both comparisons) and resulted in 11.8% and 16.3% higher elastic energy return compared to use of the Catapult FX6 (p = 0.016) and Cheetah Xtend (p<0.001) RSPs, respectively.

Hysteresis (H) was negatively correlated with maximum speed across all RSP configurations (Fig 5C):

$$Maximum\;speed\;(m\cdot s^{-1})=-0.52\times H+11.55;\;(R^{2}=0.572,p<0.001),$$ (Eq 6)

We found that based on the equations of Beck et al. [20], the Cheetah Xtend RSPs had 17.6% less hysteresis than the 1E90 Sprinter RSPs (p<0.001), which in turn had 25.5% less hysteresis compared to the Catapult FX6 RSPs (p<0.001).

## Discussion

Contrary to our first hypothesis, alterations in prosthetic stiffness alone did not affect maximum sprinting speed for athletes with bilateral transtibial amputations. Our results agree with and extend the findings of Beck et al. [5] who reported that the effects of prosthetic stiffness on running biomechanics are attenuated at progressively faster speeds

Contrary to our second hypothesis, altering prosthetic height alone by ±0.02 m did not affect maximum sprinting speed for athletes with bilateral TTAs. A ±0.02 m change in prosthetic height is approximately a ±2% change in leg length, which could potentially change running speed by ±2% for athletes if contact time and aerial time remain unchanged [34, 35]. We used Δh = ±0.02 m, and moment of inertia and mass values derived from Baum et al. [36] to calculate that the overall moment of inertia of the leg about the hip during the swing phase would change by ±1.4% (Cheetah Xtend) and ±1.5% (1E90 Sprinter) for each J-shaped RSP. To our knowledge, there are no published moment of inertia values for the C-shaped Catapult FX6 RSPs; it is likely that there would be a similar change in the overall moment of inertia for this model. An increased moment of inertia of the RSP, and therefore of the leg, requires greater knee and hip joint torques to apply the same angular accelerations (i.e. maintain the same kinematics of the leg). Sprinters with bilateral TTAs may not be able to overcome the greater moments of inertia with taller prosthetic configurations, and thus must decrease step frequency. Ropret et al. [37] increased the moment of inertia of the legs of non-amputees by adding external masses and found that maximum running speed was reduced by 12.8% when a 1.8 kg mass was fastened just above the ankle of each leg. That reduction in maximum sprinting speed was associated with a reduction in step frequency, while step length remained unchanged. We found a non-significant trend for a negative correlation between prosthetic height and step frequency (f_step_ = 4.39−0.026×Δh; p = 0.078). This trend is supported by the findings of Beck et al. [5] who found that for every 2 cm increase in prosthetic height, step frequency decreased by 0.021 Hz for sub-maximal (3 to 9 m·s^-1^) speeds. Our findings challenge the IPC regulations that limit prosthetic height for athletes with bilateral TTAs [31]. A recent update to the IPC regulations [9] further limits the maximum allowable height for athletes with bilateral TTAs compared to the previous regulation: for example, an athlete’s maximum allowable standing height of 1.85 m according to the previous rule (35) is currently reduced to 1.71 m. This has forced athletes with bilateral TTAs to significantly modify their RSP configurations, which incurs a financial burden, and adapt their running biomechanics and training. In light of our findings that RSP height does not affect maximum speed, we encourage an open discussion on rules and classifications based on experimental data and not (only) on theoretical assumptions [7, 9].

Our third hypothesis was supported. Similar to previous studies of non-amputee sprinters [12, 13] and sprinters with unilateral and bilateral transtibial amputations [3–5], we found that shorter ground contact times (t_c_), higher stance-average vertical ground reaction forces (GRF_avg,z_), and longer contact lengths (L_c_) were associated with faster maximum sprinting speeds, indicating that these biomechanical variables likely have similar associations with sprinting performance for both non-amputees and sprinters with bilateral TTAs. Contact times for sprinters with bilateral TTAs across RSP configurations (0.116 ± 0.012 s) were similar to those reported for non-amputees [12] (0.107 ± 0.003 s, t-test: p = 0.393) and to those of the affected leg of sprinters with unilateral TTAs [3] (0.119 ± 0.011 s, t-test: p = 0.184) at corresponding maximum speeds (present study: 9.1 ± 0.9 m·s^-1^; non-amputees [12]: 9.3 ± 0.4; sprinters with unilateral TTAs [3]: 8.8 ± 1.0 m·s^-1^). Stance average vertical ground reaction forces for sprinters with bilateral TTAs across RSP configurations (1.90 ± 0.15 BW) were lower than those reported for non-amputees [12] (2.14 ± 0.08 BW, t-test: p<0.001), but similar to those of the affected leg of sprinters with unilateral TTAs [3] at corresponding maximum speeds (2.02 ± 0.12 BW, t-test: p = 0.061). Contact lengths for sprinters with bilateral TTAs across RSP configurations (1.05 ± 0.06 m) were longer than those reported for non-amputees [12] (0.99 ± 0.08 m, t-test: p = <0.001), but similar to those of the affected leg of sprinters with unilateral TTAs [3] at corresponding maximum speeds (1.04 ± 0.07 m, t-test: p = 0.672).

We found that faster maximum speeds are associated with increased vertical stiffness for all of the prosthetic configurations tested in sprinters with bilateral TTAs. This is similar to what previous studies report for non-amputees [18] and athletes with unilateral and bilateral TTAs [4]. Increased vertical stiffness is the result of increased vertical ground reaction force and decreased vertical displacement of the center of mass at faster maximum speeds. A post-hoc analysis of our results indicates that decreased vertical displacement of the center of mass (Δz in m) is associated with faster maximum speeds for all of the prosthetic configurations (Maximum speed = −135.05Δz+12.43, p<0.001). Our results are in agreement with the findings of McGowan et al. [4] that athletes with bilateral TTAs reduce Δz by reducing their vertical landing velocity, as indicated by a reduction in aerial times at faster maximum speeds. According to the spring mass model [34, 38], athletes could also decrease Δz by increasing the angle of their leg at touch down (θ, in radians) relative to vertical. A post-hoc analysis of our results indicates a positive correlation between θ and maximum speed (Maximum speed = 3.46 θ+7.38, p = 0.020). These findings suggest that increased vertical stiffness is associated with faster maximum speeds for all of the prosthetic configurations in athletes with bilateral TTAs and increased vertical stiffness results from increasing peak vertical force, reducing aerial time, and increasing the angle of the leg at touch down.

We found that decreased leg stiffness is associated with faster maximum speeds for all of the prosthetic configurations in sprinters with bilateral TTAs. Previous studies of non-amputees report contrasting findings regarding leg stiffness and running speed. While some studies found no relationship [19], others found a positive correlation between the two variables [39]. Hobara et al. [40] reported that runners with unilateral TTAs had significantly greater unaffected leg stiffness (k_leg_) compared to the affected k_leg_, and the values were constant for running speeds between 2.5 and 3.5 m/s. McGowan et al. [4] reported a positive correlation between dimensionless leg stiffness (K_leg_) and relative sprinting speed in non-amputees, but a negative correlation for the affected legs of sprinters with unilateral and bilateral TTAs. Beck et al. [5] also report a negative correlation between leg stiffness (k_leg_) and absolute running speeds between 3 and 7 m·s^-1^ for athletes with bilateral TTAs. Both studies [4, 5] found an increase in the peak compression of the leg (ΔL) at progressively faster speeds in sprinters with bilateral TTAs that, given a correspondingly smaller increase in peak vertical force, leads to an overall decrease in leg stiffness. A post-hoc analysis of our results indicates that faster maximum speeds are associated with increased ΔL, in m, (Maximum speed = 12.35ΔL+7.07, p = 0.013). This, in combination with decreased vertical displacement of the center of mass (Δz), indicates that faster maximum speeds are associated with increased peak leg compression across all RSP configurations in athletes with bilateral TTAs. Increased peak leg compression is associated with an increased angle of the leg at touch down (θ), similar to what Beck et al. [5] reported for sub-maximal speeds (3–7 m·s^-1^). Our linear mixed model did not evidence a direct association between the angle of the leg at touch down and maximum speed. However, there is a clear relationship between θ, leg length (L_0_) and contact length (L_c_) (L_c_ = L_0_sin(θ)) [34, 41, 42]. An increase in the angle of the leg at touch down is represented in our model by a corresponding increase in contact length and reflects a similar positive correlation evidenced by Beck et al. [5] at slower speeds (3–7 m·s^-1^). These findings indicate that the association of faster maximum speeds and decreased leg stiffness in athletes with bilateral TTAs is associated with an increased angle of the leg at touch down.

We found that increases in step length and step frequency were associated with faster maximum speeds for all of the prosthetic configurations in sprinters with bilateral TTAs. Previous research on non-amputee sprinters [10] and sprinters with unilateral TTAs [3] also found that both step length and step frequency increase at faster speeds. Our results are in accord with and extend our previous study [5], which found that athletes with bilateral TTAs increase both step length and step frequency when running from slow (3 m·s^-1^) to progressively faster (up to 9 m·s^-1^) speeds for any given RSP configuration.

Use of the two J-shaped RSP models that resulted in the fastest maximum speeds, the Cheetah Xtend and 1E90 Sprinter RSPs, was associated with all of the biomechanical parameters associated with maximum speed except for aerial time and step frequency. At maximum speed, the use of both RSP models resulted in longer contact lengths, lower leg stiffness, and longer step lengths compared to use of the Catapult FX6 RSPs. In addition, maximum speeds were associated with different biomechanical variables for the J-shaped RSPs compared to the C-shaped Catapult FX6 RSPs. In particular, at maximum speed use of the Cheetah Xtend RSPs resulted in shorter contact times and higher stance average vertical GRFs, while use of the 1E90 Sprinter RSPs resulted in lower vertical stiffness, compared to the C-shaped Catapult FX6 RSPs. Other factors such as different sagittal plane alignment, the width, thickness and geometry of each RSP model, and the RSP moment of inertia may elicit different biomechanics that are associated with faster maximum speeds.

We accept our fourth hypothesis that the use of the prosthetic configuration that results in the fastest maximum speed maximizes the energy return per step. Lower hysteresis values in J-shaped RSPs compared to C-shaped RSPs, as shown by Beck et al. [20], allow greater elastic energy return (E_RSP_) and mechanical power return (P_RSP_). Our results indicate that faster maximum speeds are associated with greater E_RSP_ and P_RSP_ when athletes with TTAs use J-shaped RSPs. Further, use of RSP models with low compared to high hysteresis values, i.e. more energy return, may elicit faster maximum speed in athletes with TTAs.

We encountered some limitations in our study. We did not find statistically significant interactions among the biomechanical variables included in Eq 1 using the linear mixed model. However, it is likely that these biomechanical variables cannot be independently changed. For example, changes in contact and aerial times are associated with the vertical ground reaction forces [12] and, in turn, vertical and leg stiffness values. We were unable to match the maximum IPC competition height for one subject with the Catapult FX6 RSPs due to his relatively long residual limb lengths, and for another subject with the 1E90 Sprinter RSPs due to his relatively short residual limb lengths in combination with the build height of the RSPs (Table 1). We re-ran our statistical analyses omitting these two specific conditions and did not find a significant association between prosthetic height and maximum sprinting speed (p = 0.993). During the alignment sessions, we ensured that, for each subject, both sets of sockets used with J-shaped and C-shaped RSPs were adjusted similarly based on the subjects’ feedback and prosthetist’s alignment, but we could not measure or control residual limb movements within the sockets. Though unlikely, the differences between sockets could have resulted in potential differences in sprinting performance. The location of the RSP attachment to the sockets, posterior for J-shaped versus distal for C-shaped models [5], and their design (Fig 1) could have introduced discrepancies such as different masses and moments of inertia that may have altered running biomechanics and maximum speed. We acknowledge that our sample size (n = 5) limits our statistical power, but along with previous data from our group [5, 24], to our knowledge this is the largest to date published dataset of athletes with bilateral TTAs. Furthermore, the magnitude of RSP stiffness and height changes used in this study may have reduced our ability to detect statistically significant effects of RSP configuration on maximum speed.

## Conclusions

Prosthetic model (shape), but not stiffness or height, is associated with maximum sprinting speed in athletes with bilateral transtibial amputations. Use of prosthetic models with a J-shaped design resulted in 8.0–8.3% faster maximum sprinting speeds compared to a prosthetic model with a C-shaped design. Among different model, stiffness and height prosthetic configurations, shorter contact and aerial times, higher stance average vertical ground reaction forces, longer contact lengths, lower leg stiffness, higher vertical stiffness, longer step lengths and higher step frequencies were associated with faster maximum sprinting speeds in athletes with bilateral transtibial amputations. Our findings that RSP height changes of ±0.02 m do not affect maximum speed, one of the key aspects of performance, are in contrast with current International Paralympic Committee (IPC) regulations that limit the competition height of athletes with bilateral transtibial amputation. Based on our findings, we encourage the governing bodies of athletics to adopt regulations based on scientific evidence.

## Appendix

We identified ground contact time (t_c_) and aerial time (t_a_) using a vertical GRF threshold of 20 N and calculated step frequency (f_Step_) as:

$$f_{Step}=\frac{1}{t_{c}+t_{a}}$$ (Eq 7)

and step length (l_step_) as:

$$l_{step}=s/f_{Step}$$ (Eq 8)

where s is treadmill speed in m·s^-1^.

We also calculated peak and stance average vertical GRFs, and peak positive and negative horizontal GRFs (in units of body weight, BW). We calculated k_vert_ as the peak vertical ground reaction force (GRF_max,z_, in Newtons) divided by the peak vertical displacement of the center of mass (Δz, in meters):

$$k_{vert}=\frac{{GRF}_{max,z}}{\Delta z}$$ (Eq 9)

and k_leg_ as the peak vertical GRF (GRF_max,z_) divided by the peak leg compression (ΔL, in meters):

$$k_{leg}=\frac{{GRF}_{max,z}}{\Delta L}$$ (Eq 10)

We calculated Δz by integrating the vertical acceleration of the center of mass twice [43]. We measured initial leg lengths (L_0_) for each trial as the distances from the greater trochanters to the most distal locations of the unloaded RSPs. We then calculated ΔL as:

$$\Delta L=\Delta z+L_{0}(1-\cos\;\theta )$$ (Eq 11)

where θ is the angle in radians of the leg at initial contact with the ground, calculated as:

$$\theta ={sin}^{-1}\left(\frac{v\times t_{c}}{2\times L_{0}}\right)$$ (Eq 12)

(see Farley and Gonzales [34], for a detailed description of Eqs 11 and 12).

We calculated dimensionless stiffness, K_vert_ and K_leg_, by multiplying k_leg_ and k_vert_ by L_0_ divided by the body weight (BW) of each subject:

$$K_{vert}=k_{vert}\left(\frac{L_{0}}{BW}\right)$$ (Eq 13)

$$K_{leg}=k_{leg}\left(\frac{L_{0}}{BW}\right)$$ (Eq 14)

Body weight included the weight of each athlete and his RSPs and was measured by averaging the vertical GRF data over 10 strides for each trial. For each RSP configuration, we calculated mechanical power (p_RSP_) and energy return (e_RSP_) during the second half of the ground contact phase as a function of prosthetic stiffness (k_RSP_), peak prosthetic displacement (Δd), prosthetic hysteresis (H_RSP_) [20], and step time (t_step_):

$$p_{RSP}=\frac{k_{RSP}({\Delta d)}^{2}(1-H_{RSP}/100)}{2t_{step}}$$ (Eq 15)

We used the equations reported in Beck et al. [20] to calculate Δd given the measured GRF_max,z_ for each trial, multiplied by 1000 and divided by the calculated displacement to obtain prosthetic stiffness (k_RSP_, kN·m^-1^), which is utilized in Eq 15 and in subsequent analyses [5].

Dividing p_RSP_ by running speed (s), equals the energy return per meter travelled:

$$e_{RSP}=\frac{p_{RSP}}{s}$$ (Eq 16)

To compare different subjects, we divided both quantities by each subject’s body mass including his RSPs (m) [24]:

$$P_{RSP}=\frac{p_{RSP}}{m}$$ (Eq 17)

$$E_{RSP}=\frac{e_{RSP}}{m}$$ (Eq 18)

where P_RSP_ is measured in W·kg^-1^ and E_RSP_ in J·kg^-1^·m^-1^.

**Appendix Table 1:** Maximum speeds resulting from each RSP model for different stiffness categories.

**Model**	**Category**	**Maximum Speed** (m/s)
1E90 Sprinter	-1	9.27 ± 0.59
	Rec	9.54 ± 0.93
	+1	9.05 ± 1.22
Catapult	-1	8.48 ± 0.80
	Rec	8.89 ± 1.05
	+1	8.68 ± 1.01
Cheetah Xtend	-1	9.04 ± 0.83
	Rec	9.54 ± 0.72
	+1	9.76 ± 1.11

Values for Maximum Speed are reported as average ± standard deviation. Rec is the manufacturer-recommended category, -1 and +1 represent one category softer and one category stiffer respectively. All 5 subjects ran using three RSP models with three stiffness categories.

**Appendix Table 2:** Maximum speeds resulting from each RSP model for different: Stiffness categories prosthetic heights.

Model	*Δh* (cm)	Maximum Speed (m/s)
1E90Sprinter	-5**	10.00
	-4***	8.25
	-3**	10.08 ± 0.38
	-2	9.08 ± 0.14
	IPC max	9.15 ± 0.90
	2	9.50 ± 0.71
Catapult	-2	8.42 ± 1.18
	IPC max	8.48 ± 0.88
	2	8.83 ± 1.44
	10*	9.67 ± 0.38
	12*	9.00
	14*	8.00
Cheetah Xtend	-2	9.15 ± 1.17
	IPC max	9.42 ± 0.84
	2	9.69 ± 0.89

Values for Maximum Speed are reported as average ± standard deviation. Δh is the change in prosthetic height in cm compared to the International Paralympic Committee maximum allowable height (IPC max). All 5 subjects ran at varied RSP heights. Asterisks mark conditions where IPC max ± 2 cm was not attainable due to RSP model geometry and residual limb anatomy (*: Subject 1, **: Subject 2, ***: Subject 3).

## Supporting information

S1 File BADER—Bilaterals top speed data. Maximum sprinting speed and biomechanical parameters for each subject in each tested condition.
(XLSX)
